The article "Our Surgical Results in Popliteal and Infrapopliteal Artery Injuries: 21 Cases without Amputation" was published in 2024. Journal: Emerg Med Int.

# Our Surgical Results in Popliteal and Infrapopliteal Artery Injuries: 21 Cases without Amputation

**DOI:** 10.1155/2024/1721047

**Published:** 2024-01-24

**Authors:** Burak Tamteki̇n, Güler Gülsen Ersoy

**Affiliations:** Department of Cardiovascular Surgery, Faculty of Medicine, Kastamonu University, Kastamonu, Türkiye

## Abstract

**Objectives:**

Popliteal and infrapopliteal artery injuries have significant morbidity and mortality rates, especially in terms of amputation. In our study, we aimed to evaluate patients who operated due to popliteal and infrapopliteal vascular injuries in our clinic. *Patients and Methods*. Between 2016 and 2023; 21 patients who were operated in our clinic due to popliteal and infrapopliteal artery injuries were retrospectively evaluated.

**Results:**

2 of the patients were female (9.5%) and 19 were male (90.5%). Age ranges were 21–78. The causes of injury were gunshot wounds in 9 patients (42.86%), blunt trauma in 7 patients (33.33%), and sharp object injuries in 5 patients (23.80%). Reversed saphenous vein interposition in 7 patients (33.33%), primary repair in 6 patients (28.57%), 6 mm polytetrafluoroethylene graft (PTFE) interposition in 3 patients (14.28%), end-to-end anastomosis in 2 patients (9.52%), saphenous-PTFE composite graft interposition in 2 patients (9.52%), and embolectomy in 1 patient (4.76%) were performed. Arterial ligation was not performed. Simultaneous orthopedic intervention was performed in 8 patients. Fasciotomy was performed in 3 patients. Venous repair was performed in 5 patients with venous injuries. Vein ligation was not performed. Mortality was observed postoperatively in 1 patient. No patient developed amputation. Foot drop developed with nerve damage in 2 patients.

**Conclusion:**

Mortality and morbidity rates may increase in popliteal and infrapopliteal artery injuries in cases of hemodynamic disorder, simultaneous bone fracture, multivessel injury, and nerve transection. These rates can be reduced by appropriate surgical repair and ensuring hemodynamic stability.

## 1. Introduction

In civilian life, the rate of popliteal artery injuries among arterial injuries is 5–10% [1]. Although this rate is low among all extremity injuries, it is important in terms of mortality and morbidity. Popliteal artery injuries are the most risky injuries in terms of amputation among all extremity artery injuries. Amputation rates are more common in popliteal artery injuries than in other artery injuries. Like all vascular injuries; appropriate and early intervention is important in popliteal and infrapopliteal artery injuries. Therefore, appropriate surgical treatment must be performed as soon as possible and before irreversible ischemia begins [2].

In this study, we evaluated our patients with popliteal and infrapopliteal artery injuries. We aimed to emphasize the importance of appropriate and early surgical intervention in terms of amputation in popliteal artery injuries.

## 2. Materials and Methods

Between 2016 and 2023, 21 patients operated in our clinic due to popliteal and infrapopliteal artery injuries. These 21 patients, who were admitted to our hospital's emergency department due to popliteal and infrapopliteal artery injuries and operated, were evaluated retrospectively. Between these dates, all patients operated on due to popliteal and infrapopliteal artery injuries were 21 patients. Therefore, all patients were included in the study.

Before the start of the study, approval was obtained from Kastamonu University Clinical Research Ethics Committee with the number (2023-KAEK-126). 2 of the patients were female (9.5%) and 19 were male (90.5%). Age ranges were 21–78. The patients were diagnosed in our emergency department by anamnesis, physical examination, and CT angiography. The causes of injury were gunshot wounds in 9 patients (42.86%), blunt trauma in 7 patients (33.33%), and sharp object injuries in 5 patients (23.80%) (Table 1).

There were popliteal artery injury in 11 patients (52.38%) and infrapopliteal artery injury in 10 patients (47.6%). There were 5 (23.8%) anterior tibial artery injury and 5 (23.8%) posterior tibial artery injuries. Additionally, 5 patients had venous injury (23.80%).

14 (66.66%) of the arterial injuries were complete arterial rupture; 6 (28.57%) were incomplete arterial ruptures. There was total arterial thrombosis in 1 patient (4.76%) without any rupture or cut in the artery (Table 2).

## 3. Statistical Analysis

Statistical analysis was performed using the Statical Package for the Social Sciences program (SPSS, 20.0). Since the number of cases in our study was low, descriptive statistics were performed. Frequencies and percentages were used for specific measurements.

## 4. Results

Reversed saphenous vein interposition was performed in 7 patients (33.33%). Primary arterial repair was performed in 6 patients (28.57%). Direct 6 mm PTFE graft interposition was performed in 3 patients (14.28%). PTFE graft interposition was completed by first performing distal anastomoses and then proximal anastomoses. End-to-end arterial anastomosis was performed in 2 patients (9.52%). Saphenous vein-PTFE composite graft interposition was performed in 2 patients (9.52%). Embolectomy was performed in 1 patient (4.76%) (Table 3).

Simultaneous orthopedic intervention was also performed in 8 patients. First, artery repairs were performed; then orthopedic interventions were performed. Fasciotomy was performed in 3 patients. Fasciotomies were performed simultaneously with artery repairs. No artery ligation was performed. In all arterial injuries, embolectomies were performed on the distal and proximal sides of the injured artery to ensure back flow and run off. Embolectomy was performed before anastomosis or repair in all arterial injuries.

Simultaneous venous repair was performed in 5 patients with venous injuries. 3 of the venous injuries were complete lacerations. End-to-end venous anastomosis was performed in these patients. The other 2 venous injuries were incomplete. In these 2 patients, the cut venous structures were repaired. Vein ligation was not performed.

Foot drop developed in 2 patients postoperatively. However, these patients were able to walk after rehabilitation.

Mortality was observed in 1 patient after surgery. This patient had previous prosthetic mitral valve surgery (MVR) and was using warfarin. This patient's below-knee popliteal artery was ruptured in the long segment as a result of a nonvehicular blunt traffic accident. Additionally, the patient had multiple fractures in the tibia and fibula (Figure 1). During the surgery, it was observed that the patient's popliteal artery had a long segment rupture due to crush injury. 6 mm PTFE graft was interpositioned in this segment (Figure 2). External fixators were placed by orthopedics. However, the patient's bleeding could not be stopped in the postoperative period. Despite all bleeding control practices and treatments and appropriate arterial surgical repair, we could not stop our patient's bleeding. We think that the cause of death in this patient was due to multiple fractures blood leakage. Because there was no leakage from our anastomoses, we lost this patient due to coagulation disorder and bleeding diathesis. Since the patient was using warfarin, coagulation bleeding was first considered. All bleeding stopping treatments and coagulant agents were given. However, no clotting was observed. The patient quickly went into hemorrhagic shock. Although amputation was considered, the patient died from hemorrhagic shock quickly before there was a chance.

Between 2016 and 2023, 21 patients were operated on in our clinic due to popliteal and infrapopliteal vascular injuries. There was no amputation in any of our patients during early and late follow-up.

## 5. Discussion

Popliteal artery injuries are the most common cause of amputation among extremity arterial injuries [3]. The popliteal artery is the true terminal artery with a weak collateral network. It is responsible for blood circulation in the calf muscle. The popliteal vein also provides most of the lower leg and foot drainage. This explains why injury to these vessels is so dangerous [4, 5].

In the presence of popliteal and infrapopliteal artery injury, vascular repair is very important in terms of mortality and morbidity. However, in the presence of hypovolemia; correction of hemodynamics is a basic requirement. The main goal before and during surgery is bleeding control [6].

Popliteal and infrapopliteal artery injuries were diagnosed in our patients by anamnesis, physical examination, and contrast-enhanced computed tomography. 8 (38%) of our patients had orthopedic fractures. Patients with blunt trauma also had bone fractures. This situation was similar to that in the literature [7]. In patients requiring orthopedic intervention, vascular intervention was first performed. Then orthopedically necessary fixators were placed. However, in each case, the vascular grafts or repaired arteries were evaluated by us for patency after orthopedic intervention.

All arterial injuries were repaired. Artery ligation was not performed to any patient. First, distal and proximal embolectomy was performed on the ruptured arteries. Thus, runflow and backflow were achieved. Then, arterial repairs were performed. It was observed that total popliteal artery thrombosis was due to blunt trauma in 1 patient. No rupture in the artery was detected in this patient. In this patient, arterial flow was established by embolectomy.

Although we performed direct 6 mm PTFE graft interposition in 3 patients and saphenous-PTFE composite graft interposition in 2 patients, we did not observe any postoperative graft infection.

Amputation rates can rise up to 30% in the popliteal artery and vein simultaneous injuries [8]. Among the factors affecting limb loss, the presence of venous injuries and intervention in these venous injuries are as important as successful arterial repair [9]. Therefore, we performed venous repair in 5 cases with venous injuries. We did not perform venous ligation in venous injuries. 3 of the 5 patients with venous injuries had complete vein rupture. We repaired them end to end. We performed primary venous repair in 2 patients with incomplete venous rupture. Because we performed venous repair in all venous injuries, our fasciotomy rates were low. Fasciotomy was performed in only 3 patients. We did not experience compartment syndrome. All fasciotomies were performed during surgery. These patients had prolonged clamp time, muscle edema, and vein injury. Circulation was relieved in these patients after fasciotomy. As in the literature, we think that performing prophylactic fasciotomy during surgery is more advantageous than performing it in the late period in terms of decompression [10]. Additionally, we harvested all saphenous grafts from the opposite leg to prevent venous return problems.

Between 2016 and 2023, 21 patients were operated in our clinic due to popliteal and infrapopliteal artery injuries. All patients were operated on urgently without waiting. 10 of them had infrapopliteal artery injury. In 5 of these, 10 patients had anterior tibial artery injury. The other 5 patients had posterior tibial artery injuries. There was no multiple artery injury. Therefore, multiple artery repair was not performed. Protective fasciotomy was performed in 3 patients during surgery. No artery or vein ligation was performed. All artery and vein injuries were repaired. All patients were given heparin during and after surgery. Appropriate antibiotics were given and no serious postoperative infections were observed. For all these reasons, we think that we did not experience amputation.

Popliteal artery injuries are the most risky injuries in terms of amputation among all extremity artery injuries. Various amputation rates are reported in the articles. In civilian practice, amputation rates display a wide range (0%–30%). [11–13]. Except for 1 patient who died, 20 patients were discharged without amputation in our series.

Like all vascular injuries, appropriate and early intervention is important in popliteal and infrapopliteal artery injuries. For this purpose, we operated on all patients within 1 hour after the necessary examinations were performed. We repaired all artery and vein injuries. We did not perform ligation on any patient, thinking that the best approach for patients should be repair.

In literature, Lim et al. reported that they operated 31 popliteal and infrapopliteal artery injuries without amputation [14]. Therefore, we can say that our results are similar with the literature.

## 6. Conclusion

Popliteal artery injuries are the most risky injuries in terms of amputation among all extremity artery injuries. The type of trauma, how it occurs, additional bone injury, and the number and condition of injured vessels are important in terms of mortality and morbidity. Amputation rates can be reduced with appropriate and immediate surgical treatment.

We think that in case of venous injury in popliteal artery injuries, venous repair should be performed instead of venous ligation. For this purpose, we have never performed artery or vein ligation. We repaired all artery and vein injuries. Bone fractures were also treated. In this sense, we did not encounter any amputation, despite amputation rates of up to 30% in the literature. Age ranges were 21–78. We believe that life without amputation is important, especially in our young patients.

Like all arterial injuries, patients with lower extremity artery injuries should be referred to the vascular surgery clinic as soon as possible. In this sense, our study emphasizes the importance of preventing amputation in popliteal and infrapopliteal artery injuries with an early and appropriate approach.

## Figures and Tables

**Figure 1:** Multiple tibia and fibula fractures causing popliteal artery injury for left leg.

**Figure 2:** Postanastomosis image of the same patient shown in Figure 1. Figure of the patient with multiple tibia fibula fractures and popliteal artery injury. In this patient, PTFE graft was interposed submuscularly from the above-knee popliteal artery to the below-knee popliteal artery.

**Table 1:** Ethology of injuries.

Ethology	*N*	%
Gunshot	9	42.86
Blunt trauma	7	33.33
Sharp object injury	5	23.80

**Table 2:** Injury types.

Injury types	*N*	Complete	Incomplete	Thrombus
Arterial	21	14 (66.66%)	6 (28.57%)	1 (4.76%)
Venous	5	3 (60%)	2 (40%)	

**Table 3:** Operation types.

Surgeries performed	Arterial (*n* : 21)	Venous (*n* : 5)
Reversed saphenous vein interposition	7	
Primary repair (with incomplete injury)	6	2
PTFE graft interposition	3	
End-to-end anastomosis	2	3
PTFE–saphenous composite graft interposition	2	
Embolectomy (with thrombus)	1	
Ligation	0	0

## Data Availability

The data used to support the findings of the study are availability from https://doi.org/10.5281/zenodo.10207747.
